The article "Analysis of the Effect of Urban Residents' Sports Consumption on GDP Growth Based on Deep Learning" was published in 2022. Journal: Comput Intell Neurosci.

# Analysis of the Effect of Urban Residents' Sports Consumption on GDP Growth Based on Deep Learning

**DOI:** 10.1155/2022/6069881

**Published:** 2022-06-29

**Authors:** Heng Gao, Yawen Zhang, Yinhong Zhao, Junjie Ma, XinGuo Yuan

**Affiliations:** ^1^College of Education and Sports Sciences, Yangtze University, Jingzhou, China; ^2^School of Physical Education and Health, Guangxi Normal University, Guilin, China

## Abstract

Nowadays, emerging industries are emerging, and the sports industry has become a remarkable new economic growth point. Vigorously tapping the potential of residents' sports consumption has important theoretical and practical significance for promoting the development of the sports industry, improving people's living standards, and stimulating economic growth. In this paper, a deep learning model is constructed, and the random forest and random network models in the deep learning network are used to analyze the pulling effect of urban residents' sports consumption on economic growth. Since the consumption level of urban residents is much higher than that of rural residents, urban residents are in a dominant position in sports consumption, so this paper takes urban residents' sports consumption as the core to explore the pulling effect of urban residents' sports consumption on economic growth. The research theme of this paper is the pulling effect of urban residents' sports consumption on economic growth, so this paper sets the explanatory variable as the added value of GDP, expressed by GDP. Sports consumption has the characteristics of inevitability, gradualness, and diversity. With the continuous change of people's living standards, sports consumption also presents several stages of relative consumption pattern changes. Research shows that sports consumption has a positive role in promoting economic growth and the transformation and upgrading of economic development mode. Every one percentage point change in sports consumption leads to an economic growth of 0.186 percentage points, and with the increase of the lag period, urban residents' sports consumption will gradually increase the driving effect of economic growth. This effect can be analyzed at the micro- and macrolevels and enhanced by a causal cumulative cycle mechanism.

## 1. Introduction

The needs in social production and life are people's desire to obtain something to satisfy their own desires under certain conditions, and it is the driving force for a series of human behaviors. Demand, defined in GDPs, is the quantity of goods that consumers are willing and able to buy in a certain period of time and at a certain price level. Then, people's demand for sports can be defined as the number of sports consumers who are willing and able to buy sports commodities at a certain market price level within a certain period of time [1]. Demand is the driving force for people to generate consumption behavior, and similarly, sports demand is the driving force for sports consumption. Sports consumption will be generated when there is a demand for sports. Sports consumption is not only affected by GDP, social, political, cultural, and environmental factors but also by people's values, lifestyles, living habits, consumption characteristics, etc. From the perspective of GDPs, the motivation of sports demand can be roughly classified into two aspects. On the one hand, it is the pursuit of immediate consumption utility. When people participate in sports activities and buy sports goods and services, they can obtain satisfaction directly from psychological or physical to varying degrees [2]. For example, participating in sports such as swimming, skiing, and yoga can relax and delight the body and mind, watching synchronized swimming and rhythmic gymnastics can bring beauty to people, and watching NBA basketball and World Cup football can make people excited and stimulated. What sports brings to consumers is an immediate benefit, which can directly enter the consumer's utility function. In addition, most participatory sports can also give people a healthy body, and health itself can be regarded as a consumption utility, and sports consumers are satisfied because of their physical comfort. On the other hand is the pursuit of future investment returns. Physical exercise can form healthy capital in human capital, and it can prolong the working hours of workers, improve work efficiency and quality, and gain an advantage in the labor market, thereby obtaining higher income [3].

The article "Analysis of the Effect of Urban Residents' Sports Consumption on GDP Growth Based on Deep Learning" was published in 2022. Journal: Comput Intell Neurosci.

Sports brings a future benefit to consumers. People are willing to take time to participate in sports activities to exercise because they expect that the effectiveness of physical exercise will be enough to make up for the monetary expenditure and opportunity cost of taking up time to participate in sports activities. Different people have different motivations to participate in physical activities, which may be related to factors such as age and experience. In general, young people may want more direct pleasure from physical activity, but as they get older, they tend to turn more interested in healthy forms of physical activity. Since the consumption level of urban residents is much higher than that of rural residents, urban residents are in a dominant position in sports consumption. This paper uses the method of deep learning to multiply the per capita sports consumption of urban residents by the annual number of urban residents to obtain the total sports consumption data of urban residents. Therefore, this paper takes urban residents' sports consumption as the core to explore the driving effect of urban residents' sports consumption on GDP growth. It has a certain reference value [4].

The research theme of this paper is the pulling effect of urban residents' sports consumption on GDP growth, so this paper sets the explanatory variable as the added value of GDP. Consumer behavior analysis is driven by data. It is necessary to filter out main factors and design features from various information such as consumers, commodities, and consumption behaviors and use machine learning algorithms to train models on the selected data to predict consumers with the trained models and buy the most likely item. The prediction method based on consumer behavior is one of the important ways to accurately recommend the Internet and improve the purchase rate of goods. At present, this method has become a research hotspot in many disciplines such as machine learning and recommender systems [5]. The core of the consumer behavior analysis and prediction problem is to construct potential data features and build a prediction model with low cost so as to achieve the purpose of increasing the transaction scale.

The chapter arrangement of this paper: the first chapter introduces the relevant scholars' research on the consumption adjustment effect of urban residents; the second chapter introduces the basic probability of deep learning and applies the random forest and deep network in deep learning to sports consumption behavior data The third chapter makes an experiment and analyzes the relationship between urban residents' sports consumption and GDP effects based on deep learning; the fourth chapter summarizes the full text.

The innovation of this paper: Relevant scholars have now fully realized the importance of sports consumption to GDP growth, but from the perspective of existing related research progress, there is a lack of research on the regional structure of sports consumption, and it is not possible to analyze sports from the perspective of regional differences the relationship between consumption and the coordinated development of regional economy. Based on this, the research content of this paper mainly studies the significance of sports consumption to GDP growth from a macroperspective and makes a specific analysis of the relationship between sports consumption and GDP effects from the perspective of deep learning.

## 2. Related Work

In view of the special significance of sports consumption to GDP growth, the research of foreign scholars mainly focuses on the following aspects: the definition of sports consumption behavior, the demand of sports consumption market and residents' expenditure, and the motivation and behavior of sports consumption.

The article "Analysis of the Effect of Urban Residents' Sports Consumption on GDP Growth Based on Deep Learning" was published in 2022. Journal: Comput Intell Neurosci.

Zhao et al., according to the contemporary sports consumption's pride that comes from favorable marketing prospects, pointed out that in the research of marketing and sports consumer behavior, the feeling and process of pride has been achieved, and although they have been very important to sports consumers and operators, marketers have a significant impact. In this article, the findings are qualitatively analyzed through a multidimensional process view, with fan capital providing pride as a factor. Targeting four types of pride, introspective, alternative, contagious, and compelling, their research experiences and results are always in development, and a range of theoretical and managerial outcomes influence the final recommendations, making sports consumer pride in a brand or company may lead to stronger commitment and loyalty, combined with increased consumption, word-of-mouth industry and collaboration to create value [6]. Xiangqian conducted a study on the 1992 Barcelona Olympics and concluded that the total GDP impact of the Barcelona Olympics between 1987 and 1992 was US$26.048 billion. The number of employment opportunities brought by the Olympic Games was 59,328 [7]. Ding and Kong summed up the qualitative and quantitative investigations of consumer behavior in their published paper. They proposed that the investigation of consumer behavior should clarify the consumer's living background, consumption motives, and consumption patterns; fully understand consumers; and then analyze consumption behavior. In the qualitative investigation, the method of group discussion is used to explore the consumer's brand cognition, purchasing habits, usage habits, and brand evaluation [8]. Ahmad and Hall used the improved behavior tree model to analyze and predict consumer behavior and compared the models before and after the improvement. The experimental results show that the improved model has improved the effect of analyzing and predicting consumer behavior, which further proves that the decision tree model is very effective and has improvement value and potential [9]. Peng and Zeng, through the analysis of impulse response function, pointed out that GDP growth has a greater impact on urban residents' sports consumption, while the impact of urban residents' sports consumption on GDP growth is relatively low in the initial stage but gradually increases with time [10]. Ali et al. work to explore the determinants of household spending when participating in sports. Due to the huge amount of data, taking a simple regression method is not suitable. Specifically, they looked at whether factors involved in decision-making (spending money) influenced parental participation in sports, household income, education, sports club membership, and frequency of exercise. These determinants (spending large amounts of money on sports participation) included household income, participation in sports when parents were young, sports club membership, frequency of exercise, youngest child, and family size. In addition, the results suggest that a two-stage approach is necessary because it provides a more in-depth look at household spending behavior. For example, highly educated families often participate in sports and invest a lot of money [11]. Zhang et al. pointed out that GDP development should be driven from investment demand to consumption demand in a timely manner, and gradually from external to internal, to cultivate consumption power, thereby driving the timely consumption of residents [12]. Jafarzadeh and He pointed out that consumption has a long-term and stable role in promoting GDP growth, and consumption should be vigorously stimulated. In particular, consumption by residents, which accounts for a large proportion of consumption, is an effective means to promote GDP development [13]. Chen and Yan-Li believe that in the short term, the role of rural residents' consumption on GDP growth is more obvious, while urban residents' consumption has a long-term and stable role in promoting GDP growth [14]. Zhang pointed out that the consumption rate has remained at a low level for many years, but the speed of GDP growth has been fast and stable, which mainly depends on exports and investment, but it is difficult to maintain GDP growth by relying on exports and investment for a long time without the strong support of consumption, and the quality of GDP growth cannot be improved [15]. Zhou established the basic model of cross-domain sports consumption and pointed out that the development space of cross-domain sports consumption is huge, which can stimulate the development of the sports industry and related GDP growth [16]. Peng et al. discussed the relationship between sports consumption and the structure of the sports industry and proposed that the current development of the sports industry should be based on the sports goods industry, and the sports fitness and entertainment industry should be the leading realistic choice [17].

The article "Analysis of the Effect of Urban Residents' Sports Consumption on GDP Growth Based on Deep Learning" was published in 2022. Journal: Comput Intell Neurosci.

To sum up, relevant scholars have now fully realized the importance of sports consumption to economic growth, but from the relevant research progress, the research content mainly studies the significance of sports consumption to economic growth from a macroperspective. Most of them focus on theoretical research and questionnaire research, and the research depth and intensity are insufficient, neglecting to examine the economic growth effect of sports consumption from a dynamic perspective, especially the research on the impact of sports consumption on economic growth from a quantitative perspective has not yet been seen. There is a lack of research on the regional structure of sports consumption and failure to analyze the relationship between sports consumption and the coordinated development of regional economy from the perspective of regional differences, and the analysis of the relevant transmission mechanism and its action mechanism is almost blank. Policy research on GDP growth needs to be improved urgently. Based on this, from the perspective of deep learning, this paper makes a specific analysis of the relationship between sports consumption and GDP effects.

## 3. Data Processing of Sports Consumption Behavior Based on Deep Learning

### 3.1. Build the Overall Framework of the Model

In this section, before exploring the traditional forecasting model, we first design the basic process of building a forecasting model as shown in Figure 1.

Building the model is done on the basis of data processing and feature engineering. Different algorithms are used for model training, and a unified evaluation standard is used to evaluate the effectiveness of the model, and then, the optimal model is selected to recommend and predict the sports consumption behavior in the sports consumption behavior subset so as to improve the accuracy of the recommendation. Logistic regression is one of the most widely used algorithms [18]. It can not only do regression analysis but also perform classification tasks. In dealing with classification problems, it adds *g*(*z*) transformation on the basis of linear regression model, and its function form is given in the following equation:

(1) $$\begin{array}{c} g\left(z\right)=\frac{1}{1+e^{-z}}. \end{array}$$

Since the logistic regression classification model is essentially a linear classification model, it has high requirements for input, requiring the target object to be linearly separable, the features are independent of each other, there are fewer default values in the features, and the continuous numerical features can be more efficient. It is suitable for use, but the features proposed in sports consumption and economic effects are not strongly correlated, and there is a complex nonlinear relationship. Therefore, this model is not used in this paper.

### 3.2. Random Forests and Neural Networks

In classification algorithms, decision tree is a very commonly used model, but the decision tree is prone to overfitting during training, and ensemble algorithms can often effectively solve the overfitting problem and improve model efficiency. Bagging is a representative of parallel ensemble learning algorithms [19]. Random forest is an extension of Bagging. It builds Bagging ensemble based on the decision tree as the basic learner and adds random attribute selection to decision tree training as shown in Figure 2.

The article "Analysis of the Effect of Urban Residents' Sports Consumption on GDP Growth Based on Deep Learning" was published in 2022. Journal: Comput Intell Neurosci.

Random forest is an improvement of Bagging in two aspects. One is to use CART decision tree as a weak learner. The other is to randomly select some sample features of nodes, and select the best feature among the random sample features to divide the left and right sub-numbers of the decision tree. Each branch in a random forest is a weak classifier. A label is predicted from the class label set and the output on the class label [20]. In the research of consumer behavior analysis and prediction random forest randomly solves the problem of overfitting of a single decision tree in the research of analysis and prediction of consumption behavior, and multiple decision trees improve the generalization ability. The feature of high parallelism is widely used in classification problems..

Training the neural network model essentially makes the predicted value approach the actual value, and the difference between the two is defined as a loss function. Assuming that the training set is the sample size, the overall loss function of the neural network model is given in the following equation:

(2) $$\begin{array}{c} h^{\left(l\right)}=\sigma \left(w^{\left(l\right)}h^{\left(l-1\right)}+b^{\left(l\right)}\right). \end{array}$$

The first term is the mean square error cost function, which aims to control the error between the model output and the target, and the second term is the weight decay term, which prevents the model from overfitting by the weight decay magnitude. When training a neural network, gradient descent is used to update the weights. The residual between the predicted value and the true value is shown in the following equation:

(3) $$\begin{array}{c} \delta^{L}=\frac{\partial }{\partial Z_{z}^{L}}\frac{1}{2}\left|y-h\left(x\right)\right|=-\left(y_{i}-a_{i}^{L}\right)f\left(z_{i}^{L}\right). \end{array}$$

Hidden layer residual is given in the following equation:

(4) $$\begin{array}{c} \delta^{l}=\left({\left(w^{\left(i\right)}\right)}^{T}\delta^{\left(l+1\right)}\right)\cdot f\left(z_{i}^{L}\right). \end{array}$$

Updating Weight Parameters Using Gradient Descent as shown in the following equation:

(5) $$\begin{array}{c} w^{l}=w^{l}-\eta \nabla_{w\left(l\right)}J\left(w,b\right). \end{array}$$

Neural network has the characteristics of self-learning and nonlinear mapping and has been widely used in pattern recognition, classification processing, and nonlinear prediction [21]. The wide application of neural networks has also found some problems. When the number of neurons is too large, overfitting is easy to occur; and with the increase of network derivatives, gradient disappearance is easy to occur, and the effect of learning will also be affected. *Problem*. In this paper, the gradient descent method is used to easily make the model fall into local minimization, which reduces the number of neurons in the hidden layer and is used to solve the problem that the feature information cannot be fully learned.

The article "Analysis of the Effect of Urban Residents' Sports Consumption on GDP Growth Based on Deep Learning" was published in 2022. Journal: Comput Intell Neurosci.

### 3.3. Model Construction

After the data preprocessing in the previous section, the training set and the test set are divided, and then, the model is built on this basis as shown in Figure 3.

The training set features are used as the input of random forest and neural network, respectively, and the corresponding samples are used as the output to train the model. Input the sample into the trained model, calculate the output value, evaluate the quality of the model prediction result, compare the performance of the model in the consumption behavior prediction problem, and analyze the reasons.

### 3.4. The Inevitability of Urban Residents' Sports Consumption and the Analysis of Consumption Structure

Urban residents are generally satisfied with the quality of life, which provides favorable conditions for the development of sports consumption. The premise of people's spontaneous sports consumption is that they have a lot of free time, a high proportion of disposable income, the awareness of obtaining health through reasonable exercise, and a strong interest in sports-related products. Only when the quality of life reaches a corresponding level, people will actively participate in sports consumption [22]. According to Maslow's Hierarchy of Needs theory, human beings live in a social environment and will generate five needs from their hearts. From the lowest to the highest, they are physiological needs, safety needs, love and belonging, respect, and self-actualization. After people have solved the problem of food and clothing, the social environment is relatively stable; the family, friendship, love, and other social interpersonal relationships are satisfied, and after obtaining a certain social status, they are respected by others, and finally, they will seek self-worth, through different ways to experience oneself, because sports is an industry that can constantly challenge the limits of human beings, so the birth of sports consumption has its inevitability and fully conforms to the laws of social development [23].

The article "Analysis of the Effect of Urban Residents' Sports Consumption on GDP Growth Based on Deep Learning" was published in 2022. Journal: Comput Intell Neurosci.

In this paper, the deep learning model is used to require the variables in the system to be stable, and then, the unit root test needs to be performed on the selected variable data first. The unit root test generally uses the Dick–Fuller test. According to the calculation process proposed in this paper, the ADF test results of urban residents' sports consumption and GDP growth variables are obtained as shown in Figure 4.

Although some nonstationary time series have a trend of showing common changes, there is not necessarily a direct causal relationship between these series, and the regression results do not actually contain practical significance, so in order to ensure the validity of the estimated results and avoid the appearance of pseudo-regression, the model data need to be tested for stationarity before regression. Stationarity means that the basic characteristics of the current sample time series and the fitted curve may remain continuous and stable for a period of time in the future. For other sample time series that can continue to be obtained in the future, we are also able to determine with certainty that its basic characteristics must be the same as the time series of the currently obtained samples. It can be seen that the stationarity of the time series is the most basic assumption for the classical regression analysis to continue. Predictions based on stationary time series may be ultimately valid. To test the stationarity of the data, firstly, it is necessary to draw a time series diagram of the data and observe the time series diagram and analyze the trend items and intercept items contained in the fitting curves described by each observed variable in the time series diagram. This is also necessary for the next step and prepare for the unit root test.

## 4. Quantitative Measurement of the Effect of Total Sports Consumption of Urban Residents on GDP Growth

### 4.1. The Causality Test of GDP Effects Based on Deep Learning

This paper uses economic effect causality to test the causal relationship between two variables. In the stationarity test in this paper, each variable is stable after one difference, so this paper uses a deep learning model composed of two variables and their lag variables to test the causal relationship between the economic effects of the four variables. If one is accepted and the other is rejected, there is a one-way causality. In this paper, the selection of the causal lag period of the GDP effect is selected by the selection criteria of the lag period of the two-variable deep learning model.

The article "Analysis of the Effect of Urban Residents' Sports Consumption on GDP Growth Based on Deep Learning" was published in 2022. Journal: Comput Intell Neurosci.

As can be seen from Figure 5, the relationship between GDP growth and sports consumption expenditure is somewhat in conflict with the theoretical analysis that sports consumption should significantly promote GDP growth. There is no deep learning causal relationship between different consumption behaviors and GDP, indicating that the correlation between rural residents' consumption and GDP growth is small. In the relationship between GDP growth effect and GDP, the GDP growth effect is the cause of the GDP effect of GDP at the 10% confidence level, that is, changes in urban residents' consumption can cause changes in GDP growth, but GDP is not the cause of GDP effect changes in GDP growth effects. There is a causal relationship between the GDP growth effect and sports consumption, indicating that there is a strong correlation between changes in urban residents' consumption expenditures and changes in sports consumption expenditures. There is no deep learning causal relationship between different sports consumption behaviors, economic growth effects, and different consumption behaviors, and there is little interaction between changes in rural residents' consumption expenditures, changes in sports consumption expenditures, and urban residents' consumption expenditures.

### 4.2. Cointegration Relationship Test of Deep Learning Model

According to the viewpoint of GDP theory, cointegration can be understood as the existence of an equilibrium force between GDP time series variables, that is, there is a mechanism to make nonstationary different variables move together in the long run, that is, if there is long-term stability between the variables' relationship (cointegration relationship), the growth rate of variables shows a common growth trend. Conversely, if these two or more variables are not cointegrated, there is no long-term equilibrium relationship between them. Cointegration theory selects the variables of the model based on whether there is a cointegration relationship between the variables, which makes the data foundation more stable and the statistical properties better. In order to examine whether there is a long-term stable relationship between urban residents' sports consumption and GDP growth, it is necessary to conduct a cointegration test, assuming a deterministic trend in the data, an intercept term in the cointegration equation, and a lag of 12, as shown in Figures 6 and 7.

As shown in Figures 6 and 7, at the 5% significant level, the null hypothesis is rejected, and there is no unit root in the residual of the equation. It shows that there is a long-term stable cointegration relationship between GDP and sports consumption. Sports consumption of urban residents is the GDP effect of GDP growth. Therefore, when external investment is impacted, GDP growth can be stimulated by stimulating domestic demand. The elasticity of this positive effect is 0.353, that is, every one percentage point change in sports consumption leads to a GDP growth of 0.353 percentage points, which proves that sports consumption of urban residents is an influential factor driving GDP growth. A lag order that is too small may not fully reflect the dynamics of the model, as potentially useful information contained in more distant lag values may be missed. When the lag order is too large, the number of parameters to be estimated in the model will increase, and the degrees of freedom will be reduced, which is more prominent in the case of small samples, and a too large lag order may bring additional estimation errors into the in the predicted value.

The article "Analysis of the Effect of Urban Residents' Sports Consumption on GDP Growth Based on Deep Learning" was published in 2022. Journal: Comput Intell Neurosci.

In econometrics, dependencies between time series variables in particular are rarely instantaneous. A common situation is that there is a time delay in the response of the dependent variable to the explanatory variable, and this time delay is called a lag. Lags play an important role in time series econometrics, and in practice, choosing an appropriate lag order requires a trade-off between the benefits of including more lags and the cost of additional estimation uncertainty. The traditional concept of sports consumption restricts consumers. The reason why most residents are reluctant to engage in sports consumption is because they have many uncertainties about their future life. Residents spend far less time on participatory sports consumption than on viewing sports consumption. It also shows that the overall sports consumption level of urban residents is moderately low. The formation of sports consumption concept is based on sports consumption demand as the premise and guides the generation of sports consumption motivation to promote the implementation of sports consumption behavior. This is a step-by-step mechanism process.

### 4.3. Analysis of Impulse Response Function of Deep Learning Model

Impulse response function describes the response of one endogenous variable to another endogenous variable, and the impact of a unit change on its future value in a specific period, and provides information such as the positive and negative directions, adjustment time delay, and stabilization process of the system response to the impact.  Figure 8 reflects the fluctuation of the impulse response function generated by the impact of one standard deviation new interest rate on the total GDP of urban residents.

It can be seen that when the total sports consumption of urban residents in this period has a positive standard deviation impact on the total GDP, GDP development immediately responds, showing a positive impact effect. The period from the first period to the fourth period increased steadily. As the income of urban residents continued to increase, relevant consumption policies were successively introduced to vigorously stimulate residents' consumption. Urban residents' sports consumption responded strongly to GDP growth. After the sixth period, it remained stable. It shows that urban residents' sports consumption has a significant impact on GDP development and is sustainable. The responses of sports consumption to various shocks are shown in Figure 9.

The article "Analysis of the Effect of Urban Residents' Sports Consumption on GDP Growth Based on Deep Learning" was published in 2022. Journal: Comput Intell Neurosci.

*Response of sports consumption to shocks from GDP*. The response of sports consumption to the shock from GDP starts to be positive, will be negative around the third period, and turn positive after the sixth period, and the impact will gradually weaken. As a part of GDP, sports consumption naturally increases with the growth of GDP, but in the long run, the impact of GDP growth shocks on government consumption expenditure alternates and gradually declines.

### 4.4. Analysis of Vector Error Correction Deep Learning Model

The vector error correction model (VEC) is an empirical test method that reflects the short-term dynamic relationship between variables. According to Granger's theorem, if there is a cointegration relationship among several first-order nonstationary variables, then these variables must have an error correction model expression. The error correction model is a special form of difference equation model between first-order single-integrated time series with cointegration relationship. It can not only preserve the long-term dynamic information of variable relationships but also ensure the validity of regression analysis. Vector error correction model is divided into bivariate bivariate vector error correction model and multivariate vector error correction model. In view of the analysis of two vectors of economic growth effect and sports consumption in this paper, bivariate vector error correction model is used to empirically test the short-term dynamic relationship between the total consumption of urban residents and economic growth. Because the long-term relationship between urban residents' sports consumption and economic growth effect has been determined, but whether there is short-term fluctuation between the two has been established, and a bivariate vector error correction model is established as shown in Figure 10.

The constant term is 0.5513, AIC and SC are both negative and small, the error correction value is 34.4980, and each equation in the model has a good fit. From the overall inspection of the model, AIC and SC are small and negative numbers, the error correction is too large, and the goodness of fit of the deep learning model is good. According to the evaluation statistics of the equation, for GDP growth in the short term, the coefficient of the first lag period of GDP is positive, the coefficient of the second lag period is negative, and the coefficient of the error correction term is negative. When the economy grows, the error correction mechanism will weaken the economy. The strength of growth, every one percentage point change in sports consumption, leads to a GDP growth of 0.186 percentage points. Through the above empirical analysis on the relationship between urban residents' sports consumption and GDP growth effect, it can be concluded that there is a stable correlation between urban residents' sports consumption and GDP development.

The article "Analysis of the Effect of Urban Residents' Sports Consumption on GDP Growth Based on Deep Learning" was published in 2022. Journal: Comput Intell Neurosci.

On the whole, urban residents' sports consumption has just been active. During this period, people's needs for sports consumption are still in the basic stage, or some people have just entered the demand for a comfortable environment, and fewer people have reached a higher level of demand. The needs of some consumers remain on meeting the general conditions of consumption, and the residents' awareness of sports consumption is reflected in the degree of dependence on the existing environment and the urgency to transform the environment. As far as the overall level of urban residents' sports consumption is concerned, there should be a demand for a higher level of sports consumption environment. Therefore, strengthening and guiding residents' awareness of environmental needs is an important way to promote the improvement of sports consumption. The news media plays an important role in improving residents' awareness of sports consumption. The combination of publicity and guidance will effectively change residents' demand concept. Starting from the demand, timely guidance can promote the development of residents' sports consumption demand to a high level. Residents should also take the initiative to integrate their awareness of consumer demand with their own consumption activities to coordinate with their own consumption levels.

## 5. Conclusions

The main purpose of this study is to study the relationship between sports consumption and GDP growth. The reason for the analysis is that through the analysis of the GDP effect mechanism of sports consumption, this paper summarizes the mechanism of sports consumption's role in regional development as GDP growth effect, industrial structure effect, regional agglomeration effect, and regional innovation effect. Every one percentage point change in sports consumption leads to a GDP growth of 0.186 percentage points, and with the increase of the lag period, urban residents' sports consumption will gradually increase the driving effect of GDP growth. Through the analysis of impulse response function, it can be seen that my country's GDP growth has a greater impact on urban residents' sports consumption, while the impact of urban residents' sports consumption on GDP growth is relatively low in the initial stage but gradually increases with time. The GDP growth effect of sports consumption is the display basis and dominant indicator of regional GDP development. The industrial structure effect of sports consumption is the resource converter of regional GDP development. The regional agglomeration effect and regional innovation effect of sports consumption are the strong driving force of regional GDP development. The GDP growth effect of sports consumption is mainly manifested in demand-driven GDP growth, and factors such as labor quality and technological level will also play a role. The development of sports consumption is accompanied by the construction of stadium facilities and supporting infrastructure, and the influx of event tourists will expand the total demand and stimulate GDP growth. Sports consumption will promote the development of the urban entertainment and fitness industry, improve the quality of laborers, and ultimately affect the long-term regional impact. Now we see a huge consumer market and development space for the sports industry, abandoning those resistance factors that are not suitable for the development of the sports economy, and gradually establishing a sports GDP system. With GDP development and people's living standards increasing, the socialization of sports is getting higher and higher, and the level of sports consumption will also increase, eventually forming a benign process of production, consumption, and reproduction, making sports consumption a new growth that promotes GDP growth.

The article "Analysis of the Effect of Urban Residents' Sports Consumption on GDP Growth Based on Deep Learning" was published in 2022. Journal: Comput Intell Neurosci.

As the economy has entered a new normal, the industrial structure has been optimized and upgraded, from investment-driven and factor-driven to innovation-driven, emerging industries have sprung up, and the sports industry has become an eye-catching new economic growth point. Because the consumption level of urban residents is much higher than that of township residents, and the sports consumption of urban residents is still dominant, the sports consumption level of urban residents is the core content of this study. Vigorously tapping the potential of residents' sports consumption has important theoretical and practical significance for promoting the development of the sports industry, improving people's living standards, and stimulating economic growth.

## Figures and Tables

**Figure 1:** Flow chart of building a prediction model.

**Figure 2:** Principle of random forest algorithm.

**Figure 3:** Model construction flow chart.

**Figure 4:** ADF test results of urban residents' sports consumption and GDP growth variables.

**Figure 5:** The causality test results of the GDP effects of each series.

**Figure 6:** Trace statistics test results.

**Figure 7:** The results of the largest eigenvalue statistic test.

**Figure 8:** Fluctuation of the response function.

**Figure 9:** Impulse response diagram of sports consumption to shock.

**Figure 10:** Estimation results of vector error correction model.

## Data Availability

The data set can be accessed upon request from the corresponding author.
